# Evaluation of Short-Term Efficacy of PD-1 Monoclonal Antibody Immunotherapy for Lymphoma by Positron Emission Tomography/Computed Tomography Imaging with Convolutional Neural Network Image Registration Algorithm

**DOI:** 10.1155/2022/1388517

**Published:** 2022-08-31

**Authors:** Jie Fang, Zhendong Chen

**Affiliations:** Department of Oncology, The Second Affiliated Hospital of Anhui Medical University, Hefei 230601, Anhui, China

## Abstract

The objective of this study was to investigate the value of PET/CT imaging based on CNN image registration algorithm in evaluating the short-term efficacy of PD-1 monoclonal antibody immunotherapy for lymphoma. 36 patients with advanced lymphoma confirmed by histology or cytochemistry and treated with PD-1 monoclonal antibody admitted to hospital were included. In addition, 38 normal controls were from healthy volunteers. All patients were treated with PD-1 monoclonal antibody intravenous infusion, and the image data were processed by CT with intelligent segmentation algorithm. Medication method: nivolumab 3 mg/kg for 2 weeks; pembrolizumab 2 mg/kg for 3 weeks; and continuous medication until tumor progression or unacceptable adverse reactions. Efficacy was evaluated every 3 cycles. Imaging examinations were performed after 3 weeks of medication to evaluate the therapeutic effect. The concentrations of IL-2, IL-7, basic fibroblast growth factor (FGF), granulocyte-macrophage colony-stimulating factor (GM-CSF), platelet-derived growth factor (PDGF-bb), and other factors in the normal control group were significantly higher than those in the advanced lymphoma patients, and the differences were statistically significant (*P* < 0.05). The PET/CT imaging automatic segmentation accuracy of the CNN image registration algorithm was greater than 81%, and 27 patients were treated for more than 3 cycles, including 1 case of partial remission (PR) (3.7%), 16 cases of stable disease (SD) (59.3%) after 3 cycles of treatment, and 10 cases of progressive disease (PD) (37%). After 6 cycles of treatment, 1 case was PR (8.3%), 7 cases were SD (58.4%), and 4 cases were PD (33.3%). Adverse reactions included fever, fatigue, gastrointestinal reactions, hypothyroidism, and interstitial pneumonia. PD-1 monoclonal antibody immunotherapy had a certain short-term effect on lymphoma.

## 1. Introduction

Lymphoma is a cancer that originates from the lymphatic system and is derived from malignant lymphocytes. Because these cells have many different properties and functions, and they can also enter various organs of the body, it is not difficult to think of lymphoid tumors from which they are derived. There are many different species and traits. Lymphoma is a general term for various tumors originating from the lymphatic system. Immunotherapy is considered to be one of the most important advances in tumor therapy. However, although better efficacy can be seen in most patients in immunotherapy, not all patients can produce long-term survival benefits, and the treatment effect of some immunogenic cancer patients is better, such as melanoma and renal cells. Because of this, it is necessary to further explore the development of antitumor immunotherapy [1]. The antitumor and anti-immune response is based on an extremely delicate and complex balance between anti-immune activation and anti-immune suppression in the tumor microenvironment. The antitumor and tumor-promoting functions of various immune-related cytokines in the tumor microenvironment will ultimately affect the fate of tumors. However, in the tumor microenvironment, high expression of suppressor depleted T cells, decreased T cell effector energy, depletion of effector cytokine energy, and decreased killing activity are persistently explored [2]. Studies have shown that a large number of T cells in the tumor microenvironment can cause exhaustion, and the exhausted T cells highly express a variety of inhibitory receptors, such as PD-1 monoclonal antibody (nivolumab/pembrolizumab) [3–5]. PD-1 is an immune test site receptor, and the ligand PD-L1 interacts to produce a variety of functions controlled by negative immune regulation [6]. Under normal circumstances, PD-1 is used to prevent and stop excessive immune responses and maintain the body's immune tolerance state; however, in tumor patients, PD-1 has a high level of loss of T-cell tumor elimination ability [7, 8]. Therefore, the depletion of T cells during the reversal process has become one of the strategies of tumor immunotherapy. It is important to choose an appropriate method to assess whether treatment at the immune test site can achieve reversal of T-cell depletion and remodeling of the body's immune state.

PET/CT is a fusion of PET and CT. PET is positron emission computed tomography, and CT refers to the common computed tomography. This imaging technique is used to diagnose diseases (often used in tumor-related diseases) by the difference in the ability of lesions to uptake radionuclide-labeled drugs. Because drugs can directly reach intracellular imaging, it is called bioimaging. Multimodal medical image registration is to register images from different medical image devices in the future, which can make full use of the characteristics of each image and complete the mutual complementation of information [9]. Medical imaging models can be divided into two categories: functional imaging is mostly used to detect the dynamic changes of human metabolism and function, such as fMRI [10], and decomposition imaging mainly shows the physiological decomposition structure features of the human body, such as X-ray, CT, and ultrasound (US) [11]. The energy images are of slightly lower resolution but can provide information on the energy metabolism of the donor organ, which anatomical images cannot. Anatomical images have high resolution and can provide information on the anatomical morphology of organs but cannot express the functional information of organs [12]. After registering the anatomical image and the functional image, the information of various aspects of the human body can be reflected on a medical image at the same time: fully display the structure, function (biochemical, physiological, metabolic process), and transformation of tissues or organs, and organically combine anatomy and function. It can provide effective data for clinical diagnosis and observation of treatment sites. In particular, the fusion of PET, CT, and magnetic resonance imaging (MRI) images has wider clinical application value and development potential [13, 14]. It can provide complete information for clinical diagnosis of complex imaging and accurate anatomy and positioning for surgical treatment. Cellular neural network (CNN) has been widely used in the field of image processing. The advantages of CNN are as follows: first, it has the characteristics of continuous time, which can meet the requirements of real-time image signal processing; second, its local interconnection feature makes it convenient for hardware implementation, especially suitable for high-speed parallel processing; and third, there is no correlation between the processing speed of CNN and the image canonical mode [15–17]. In this study, the short-term efficacy of PD-1 monoclonal antibody immunotherapy in the treatment of lymphoma was evaluated using PET/CT imaging with CNN image registration algorithm.

## 2. Materials and Methods

### 2.1. Research Subjects

Thirty-six patients with advanced lymphoma who were histologically or cytochemically confirmed and treated with PD-1 monoclonal antibody who were admitted to hospital from February 2019 to December 2020 were included. 38 normal controls were from healthy volunteers. In the PD-1 treatment group, the patients' age range was 36–89 years, including 20 men and 13 women. The control group included 10 men and 25 women, aged 26–57 years. This study was approved by the ethics committee of the hospital, and the families of the patients participating signed the consent form.

Inclusion criteria were as follows: patients received immunotherapy with PD-1 monoclonal antibody, and patients who voluntary the treatment study. Exclusion criteria were as follows: patients with severe organ dysfunction, and investigators who were unwilling to accept treatment.

### 2.2. Inspection Methods and Evaluation Indicators

Whole-body F-FDG PET/CT scanning was performed. The head scan was performed first, and the scan range was from the top of the skull to the submental level. Parameters were set as follows: spiral CT, tube voltage 124 kV, tube current 382 mA, 0.9 s/rot; and PET, 3D acquisition, single bed, time 4 min. Afterward, a body scan was performed, and the scan range was from the base of the skull to the upper middle and upper thighs. Parameters were set as follows: spiral CT, tube voltage 124 kV, automatic adjustment of tube current, 0.9 s/rot; and PET, 3D acquisition, 4 to 7 beds, 3 min per bed. Attenuation correction was performed on PET images with CT images, reconstruction was performed iteratively, and image fusion was performed on workstation.

### 2.3. Artificial Intelligence Algorithm to Segment Images

Mutual information was a measure in information theory. Image mutual information registration introduces concepts in information theory, such as joint entropy and mutual information, which can make the registration accuracy reach subpixel high precision. The two medical images to be registered were defined as a floating image *U* and a reference image *D*, which were two sets of random variables with respect to the grayscale of the images. For the floating image *U* and the reference image *D*, the entropy and joint abstraction are as follows:

(1) $$\begin{array}{c} \begin{array}{c} G\left(U\right)=-\underset{u}{\sum }\;j_{U}\left(u\right)\log_{2}\;j_{U}\left(u\right),\\ G\left(D\right)=-\underset{d}{\sum }\;j_{D}\left(d\right)\log_{2}\;j_{D}\left(d\right),\\ G\left(U,D\right)=-\underset{u,d}{\sum }\;j_{UD}\left(u,d\right)\log_{2}\;j_{UD}\left(u,d\right). \end{array} \end{array}$$

The calculation expression of mutual information value is as follows:

(2) $$\begin{array}{c} I\left(U,D\right)=G\left(U\right)+G\left(D\right)-G\left(U,D\right)=\underset{u,d}{\sum }\;J_{UD}\left(u,d\right)\log_{2}\;\frac{J_{UD}\left(u,d\right)}{J_{U}\left(u\right)\cdot P_{D}\left(d\right)}. \end{array}$$

The relationship between mutual information and entropy can be expressed by the following equation:

(3) $$\begin{array}{c} I\left(U,D\right)=\left\{\begin{array}{c} G\left(U\right)+G\left(D\right)-G\left(U,D\right),\\ G\left(D\right)-G\left(U\;|\;D\right),\\ G\left(D\right)-G\left(D\;|\;U\right). \end{array}\right) \end{array}$$

The method of using mutual information needed to calculate the probability distribution of the image. The joint probability distribution of A and B is as follows:

(4) $$\begin{array}{c} J_{UD}\left(u,d\right)=\frac{n_{u\;d}}{N}, \end{array}$$

where *N* is the total number of adjacent and different grayscale pixel pairs in the edge image and *n*_*ud*_ is the number of *u*, *d* pixel pairs in the grayscale.

The independent rate distribution of *u*, *d* is as follows:

(5) $$\begin{array}{c} J_{U}\left(U\right)=\underset{d}{\sum }j_{UD}\left(u,d\right),j_{D}\left(d\right)=\underset{u}{\sum }j_{UD}\left(u,d\right). \end{array}$$

In the PET/CT image registration method based on CNN and mutual information, the signal-to-noise ratio (SNR) and spatial resolution of PET images were relatively low, the edges were blurred, and the amount of image information was less, so it was difficult to extract the edges of PET images. CT images had clear bones and high resolution, which can serve as a good reference for the localization of lesions, and edge lifting was easy to achieve. Then, the mutual information registration of the PET image and the CT edge image was performed, and finally, the fusion of the PET and CT images was realized, so that the high metabolic area in the PET image can be accurately located. Image registration based on mutual information can be expressed by the following equation:

(6) $$\begin{array}{c} u^{*}=arg\;m\left(U,D\right). \end{array}$$

where *u*^*∗*^ is the transformation parameter for the image to be registered; *U* represents the image to be registered; and *D* represents the reference image.

When two images based on a common anatomical structure achieved the best registration, the mutual information value of their corresponding pixels should be the maximum value. At this time, the corresponding optimal transformation parameter was *u*^*∗*^, and *u*^*∗*^ was obtained through the optimization search process of the mutual information function. The PET and CT images used in this study were obtained at the same time in PET/CT equipment. Therefore, it was assumed that the affine transformation relationship was satisfied between the two images to be matched.

(7) $$\begin{array}{c} \left[\begin{array}{c} x_{U}\\ y_{D} \end{array}\right]=\left[\begin{array}{c} \cos\;\beta -\sin\;\beta \\ \sin\;\beta \;\cos\;\beta \end{array}\right]\left[\begin{array}{c} x_{U}\\ x_{D} \end{array}\right]+\left[\begin{array}{c} x\\ y \end{array}\right], \end{array}$$

where *β* is the rotation angle between the two images and *x* and *y* are the translations of the pixels on the image in the *x* and *y* directions, respectively.

According to the obtained transformation parameters, the image to be registered was subjected to geometric transformation and interpolation processing, and the obtained image was the registered image. The schematic diagram of the two-dimensional cellular neural network based on the CNN image registration algorithm is shown in Figure 1.

### 2.4. Treatment Method and Effect Evaluation

All patients received PD-1 monoclonal antibody intravenous drip therapy. The medication method was as follows: nivolumab 3 mg/kg for 2 weeks; pembrolizumab 2 mg/kg for 3 weeks; and continuous medication until tumor progression or unacceptable adverse reactions. Efficacy evaluation was performed every 3 cycles. All patients underwent cytokines, blood routine, CT, and other related tests before receiving PD-1 monoclonal antibody therapy to evaluate the condition. Imaging examinations were performed after 3 weeks of medication to evaluate the therapeutic effect.

According to the RECIST solid tumor criteria, the objective response rate was divided into complete remission (CR), partial remission (PR), stable disease (SD), and progressive disease (PD).

### 2.5. Statistical Methods

SPSS16 software was adopted to complete the statistics, the measurement data were represented by $\bar{x}$ ± *s*, and the count data were represented by frequency or percentage (%). Correlations between different data were analyzed using Kappa. *P* < 0.05 was considered statistically significant.

## 3. Results

### 3.1. Basic Data

The 35 control subjects in this study were all healthy individuals with physical examination, ranging in age from 26 to 57 years, with a median age of 39 years. There were 10 males and 25 females. The PD-1 treatment group included patients aged 36 to 89 years, with a median age of 53.5 years; and there were 20 males and 13 females. The two groups of experimenters were comparable (*P* > 0.05). The specific data are shown in Table 1.

### 3.2. Evaluation of CT Image Segmentation Effect Based on Artificial Intelligence Segmentation Algorithm

As illustrated in Figure 2, the PET/CT image registration method based on CNN and mutual information combined the advantages of the two image registration methods with features and mutual information and had a relatively small relative computational time and space. Compared with the traditional algorithm, the CNN algorithm improved the speed of image registration. The automatic segmentation accuracy of the CNN algorithm was greater than 81%, the reconstruction accuracy of multidimensional organs can be observed at random angles, and the reconstruction accuracy was not lower than the original input CT resolution. The computational error of the CNN algorithm was less than 8.9%. The evaluation method of CT image segmentation effect based on artificial intelligence segmentation algorithm was the clarity of the image and the speed of image registration. Figures 2(d) and 2(e) are the results of segmentation of the target area in the CT image about the lymphatic CT image and the algorithm, and the next to the right is the enlarged image.

### 3.3. Comparative Analysis of Initial Serum Cytokine Concentrations in Normal Population and Patients with Advanced Lymphoma

The results showed that the concentrations of IL-2, IL-7, basic FGF, GM-CSF, and PDGF-bb in the normal control group were significantly higher than those in the advanced lymphoma patients, showing statistically significant differences (*P* < 0.05), as shown in Figure 3(a). The initial plasma concentration of tumor patients was significantly higher than that of normal controls. The initial serum concentrations of IL-5, IL-6, IL-8, and IL-15 in the normal control group were significantly lower than those in the tumor patients, and the difference was statistically significant (*P* < 0.05). Other cytokine concentrations were not significantly different, as shown in Figure 3(b).

### 3.4. Efficacy Changes in Lymphoma Patients during PD-1 Treatment Cycles

For 36 patients who received PD-1 treatment, serum and cytoplasmic factor tests were performed before each cycle of treatment, and 9 patients developed symptoms of disease progression after 1 to 2 cycles of treatment. 27 patients were treated for more than 3 cycles, including 1 PR (3.7%), 16 SD (59.3%), and 10 PD (37%) after 3 cycles of treatment. 17 patients who developed PR and SD after PD-1 therapy continued to receive PD-1 therapy. Among them, 12 patients were treated for more than 6 cycles, and 1 patient had PR (8.3%) when re-evaluated after 6 cycles of therapy. There were 4 cases of SD (58.4%) and 4 cases of PD (33.3%). The specific results are shown in Figure 4.  Figure 4(a) is the efficacy of 3 cycles of PD-1 treatment, and Figure 4(b) is the efficacy of 6 cycles of PD-1 treatment.

### 3.5. Changes in Serum Cytokine Concentrations during Each Cycle of PD-1 Treatment

According to the evaluation results, 12 patients were divided into PR + SD group and PD group. The dynamic changes of cytokines were analyzed (in the early morning of each cycle treatment), and the results were summarized as follows: in the PR + SD group, IL-2, IL-5, IL-15, and GM-CSF wave amplitudes were very large, but there was no upward or downward trend observed overall, while IL-7 showed a slight upward trend; and the basic FGF changed slightly more; and in the PD group, IL-2, IL-5, and IL-15 showed small overall fluctuation range; IL-7 and GM-CSF changed slightly, the overall level of basic FGF was higher, and the change range was large. The specific results are shown in Figures 5 and 6.

### 3.6. Adverse Effects

Notable adverse reactions observed in this study were pyrexia, fatigue, gastrointestinal reactions (nausea and vomiting), hypothyroidism, and interstitial pneumonia, as shown in Figure 7. The cytokines in patients with adverse reactions were analyzed, and there was no obvious correlation between the occurrence of adverse reactions and changes in cytokines. This may be due to the small number of cases and the atypical adverse reactions in some patients.

## 4. Discussion

The occurrence and development of tumors are closely related to the inflammatory and immune status of the body, and cytokine levels can reflect the inflammatory and immune status of acquired cells [18]. Cytokines are biological indicators. During the treatment, cytokine levels can change with tumor development and progression, reflecting the inflammatory disease and the corresponding state of acquired immune cells in patients. In this study, it was found that PD-1-treated patients with advanced tumors had lower IL-2 concentrations than normal groups. This may further indicate that IL-2 has an antitumor effect, and the changes in its concentration may be related to the short-term therapeutic effect of PD-1. Elevated IL-2 concentrations may indicate a better treatment effect with PD-1. Models still need to be tested and validated, and research results in this study were similar to previous studies [19, 20]. IL-5 induces immunoglobulin secretion and has antitumor activity. This study found that, during the 3-week treatment process, the PR + SD group showed a continuous upward trend, while the PD group showed a slight downward trend, which may explain the antitumor effect of IL-5. In the follow-up patients, the amplitude of the PR + SD group was higher than that of the PD group, and the amplitude of the PD group was the lowest. This may indicate that the immune response of PD patients to IL-5 is less sensitive to PD-1 treatment, which may further illustrate the antitumor effect of IL-5. In addition, changes in IL-5 concentration may be related to the short-term therapeutic effect of PD-1, and the increase in concentration may indicate a better therapeutic effect of PD-1, which needs to be studied by large-scale clinical experiments. Endodermal growth factor (VEGF) is a protein that selectively promotes the division of endodermal cells in the blood vessels and is one of the core substances that mediate angiogenesis and angiogenesis [21]. VEGF can increase the permeability of endothelial cells and facilitate the growth and migration of endothelial cells, it can be used to form a special blood-stimulating tube inner surface, and it can be associated with the formation of hematoma and gonorrhea. Excessive use of VEGF is associated with the occurrence of various tumors.

In the above discussion, the function and morphological regularity of each cell in the process of tumorigenesis and development is briefly explained. Observing the changing trends of IL-2, IL-15, IL-6, and IL-8 during PD-1 treatment may be of great significance for predicting the efficacy of PD-1. It summarized the cytokine numbers for 3 cycles and 6 weeks of treatment. It can be found that there was a trend of cytokine changes throughout the treatment process, and the change trends of different treatment effect groups (SD group/PD group) were different. Therefore, monitoring the movement of peripheral blood cells during treatment can be used to predict the therapeutic effect of TD-1 and its toxic side effects. In the course of clinical treatment, the increase of cytokines such as IL-2 and IL-15 can indicate a reasonable effect of PD-1 treatment, which is sustainable. Elevated levels of IL-6 and IL-8 may indicate a poor therapeutic effect of PD-1, which requires close observation. Furthermore, the mechanisms of cytokines are very complex and not fully understood [22]. This study only focused on the analysis of single cytokine changes. But each cell is located in a complex network, so it needs to detect as many relevant disease-free factors as possible and observe the changing trend of multiple cells [23], so as to be able to predict the efficacy of free treatment. In terms of adverse reactions, previous studies believed that anti-PD-1 monoclonal antibody treatment was safe and had a low incidence of adverse reactions. The number of cases included in this study was small, and there was a certain bias [24]. In the analysis of the observed adverse effects, there was no clear correlation between adverse effects and cellular transformation. There is still a need to further explore prospective bedside studies with large samples. A new method for PET/CT image registration based on CNN and trust information is proposed. The purpose of applying CNN to medical image registration is to use the parallel processing characteristics of cellular neural networks to improve the speed of medical image registration. The purpose of preserving mutual information image registration is to exploit the better robustness of mutual information image registration [25]. The research results show that it is an effective and feasible idea to combine multiple features with the image element similarity method, and it is proved that the advantages of the two complement each other. The sample size of this study was small and was used as a preliminary study to explore the nature of the study. It is currently believed that the changes in the concentration of some peripheral blood cytokines may be related to the efficacy of PD-1 immunotherapy. Further large-sample prospective clinical studies were needed for validation.

## 5. Conclusion

The results of this study confirmed that the changes in the concentration of cytokines in peripheral blood may be related to the efficacy of PD-1 immunotherapy, and the CNN algorithm used in the segmentation of PET/CT images of lymphoma patients can effectively improve the segmentation effect. However, in this study, the sample size was small, and more experimental people should be included. In addition, clinical trials should not be conducted in a single area or a small area and should be conducted in a multicenter, large-sample hospital. In conclusion, the results of this study can provide a reference for the early diagnosis of lymphoma and the selection of clinical treatment methods.

## Figures and Tables

**Figure 1:** Schematic diagram of the two-dimensional cellular neural network.

**Figure 2:** The result of segmentation of target area in CT image by lymphatic CT imaging map and algorithm: (a) speed of image registration between the traditional algorithm and the CNN algorithm; (b) comparison of the segmentation accuracy of the traditional algorithm and the CNN algorithm; (c) calculation error between the traditional algorithm and the CNN algorithm was less than 8.9%; and (d, e) the results of segmenting the target area in the CT image of the lymphatic CT image and the algorithm, and the right side is the enlarged image.

**Figure 3:** Comparison of initial cytokine concentrations between the two groups: (a) concentration of cytokines in the normal control group was higher than that of patients with advanced lymphoma; (b) concentration of cytokines in the normal control group was lower than that of patients with advanced lymphoma. ^∗^Compared with normal control group, *P* < 0.05.

**Figure 4:** Analysis of the efficacy of PD-1 treatment for 3 cycles and 6 cycles: (a) 3 cycles and (b) 6 cycles.

**Figure 5:** Changes of serum cytokine concentrations in the PR + SD group.

**Figure 6:** Changes of serum cytokine concentrations in the PD group.

**Figure 7:** Adverse reactions of patients.

**Table 1:** Basic data of patients.

Item	Control group	PD-1 treatment group
Age range (years old)	26–57	36–89
Median age (years old)	39	53.5
Male/female (cases)	10/25	20/13

## Data Availability

The data used to support the findings of this study are available from the corresponding author upon request.
